This article has been retracted.

# Construction of Teaching Supervision System of Applied Undergraduate Colleges and Universities under the Perspective of “Internet+”

**DOI:** 10.1155/2022/9277583

**Published:** 2022-06-22

**Authors:** Songfeng Zhang, Fucha Zhao

**Affiliations:** Guangzhou College of Technology and Business, Guangzhou 528137, Guangdong, China

## Abstract

With the wide application of “Internet +” in education and the transformation and development of applied colleges and universities, teaching supervision is an important part of colleges and universities' teaching quality assurance system. However, there are still the following problems in the actual teaching supervision. The first is emphasizing “theory” teaching rather than “practice” teaching; the second is unstable supervisory team; the third is emphasizing “supervision” rather than “guidance”; the fourth is single ways and methods of teaching supervision; the fifth is lack of integration of teaching evaluation information. In order to ensure that the teaching quality of applied undergraduate colleges and universities can meet the requirements of local social development, teaching supervision work must be rooted in reality and focused on the future to build an effective teaching supervision system. Therefore, six suggestions are put forward. The first is to attach importance to the practicality of teaching, that is, application. The second is to insist on the part-time subjectivity of the supervision team. The third is to form a supervision culture of “guidance as to the main focus, supervision as the supplement, combination of supervision, and guidance to promote teaching quality through feedback.” The fourth is to implement a triple superposition of regular supervision, inspection supervision, and special supervision. The fifth is to strengthen the synergy and innovation of supervision methods. The sixth is to establish an information-based teaching supervision and management platform so as to solve the deficiencies of the teaching supervision system in application-oriented colleges and universities in function, organization, culture, methods, methods, technology, and so on.

## 1. Introduction

At present, China is in a critical period of deepening the reform and quality construction of higher education, and it is also a key stage to accelerate the development of high-level undergraduate education and internal connotation. In 2018, the Ministry of Education issued a circular to eliminate “poor quality classes” and create “high-quality classes,” striving to improve undergraduate education and teaching. Universities have carried out undergraduate education work and great discussions on ideas, setting off the tide of quality construction. The teaching supervision system is an important guarantee for monitoring the quality of talent training in colleges and universities. It plays an important role in ensuring the quality of teaching in colleges and universities, promoting the construction of the teacher team, promoting the construction of teaching and learning styles in colleges and universities, and providing advice and suggestions for the development of schools. At present, some local universities are in a period of “transformation.” Although they have established the cultivation goal of application-oriented talents, due to the lag of education and teaching management, the uneven construction of information technology, “Internet+” technology has not been effectively used in the supervision work of universities, and there are a series of problems in the supervision system of universities in general. For example, it emphasizes the supervision of “theoretical courses” rather than “practical courses”; the supervision team is unstable; it emphasizes “supervision” rather than “guidance”; the methods and approaches are single and simple and lack technical support. To a certain extent, this has hindered the idea and correct guidance of the cultivation of applied talents in teaching, thus failing to ensure the quality of the cultivation of applied talents, and is not conducive to the development of innovation and entrepreneurship education and the integration of industry, education, and research. Therefore, giving full play to applying “Internet+” technology in teaching supervision, innovative teaching management, and building an effective teaching supervision system have become important themes and inevitable trends in the reform and development of teaching management in universities.

## 2. Importance of Teaching Supervision Work

Undergraduate teaching is the key issue that the university way should grasp. “We must place undergraduate education at the core position of building a strong country of higher education, the key position of training socialist builders and successors, and the pioneering position of national prosperity and national rejuvenation to understand and promote. We should systematically plan and promote it in terms of ideas, concepts, standards, models, culture, and systems, establish educational confidence, reflect Chinese characteristics, pursue world-class, and form a Chinese program for high-level undergraduate education” [1]. This is the speech made by Minister Chen Baosheng at the launch of the Six Excellence and One Top Notch Plan 2.0. Undergraduate education is based on undergraduate teaching, and there is no way to talk about undergraduate education without teaching. The quality of undergraduate teaching requires assurance through teaching supervision, which means that teaching supervision is significant for strengthening undergraduate teaching.

### 2.1. Ensure the Orientation of School Running

Applied universities emphasize the social service function of universities, oriented to service development needs, and focus on professional knowledge, professional skills training, and training to cultivate application-oriented talents as the goal [2]. At present, China's applied universities and local universities lack the awareness of serving the local area and the level of service. Consequently, the deviation of the insufficient concept of serving the local economy in teaching should be corrected through teaching supervision work, and the concept of serving the local area should be established. Furthermore, it relies on various local resources, integrates into local economic development, cultivates high-quality applied talents rooted in the local area, and delivers a certain quantity and quality of professional talents to the local area. In this way, it ensures the sustainable development of the local economy and provides a constant source of power and resources for the universities to meet the needs of local economic and social development.

### 2.2. Assist in Optimizing the Construction of Teaching Staff

Teachers in applied colleges and universities are responsible for serving local economic development and cultivating applied talents. In addition to solid professional knowledge, a high level of scientific research, and teaching ability, teachers should also have the practical ability to operate skillfully and have excellent technical skills. By monitoring and guiding teachers throughout the teaching process, the teaching supervision work can promptly identify the problems in the teaching process of teachers, especially the phenomenon of emphasizing theoretical teaching and ignoring practical teaching among teachers. It should give teachers helpful evaluation, targeted guidance, and intentional guidance for cultivating “dual-teacher” and “dual-competent” teachers in applied colleges and universities to optimize teachers' construction.

### 2.3. Promote the Construction of Teaching and Learning Styles in Universities

The teaching and learning style of a school is an important reflection of the spirit of teachers and students in a university. “Emphasis on academics rather than teaching” has always been a common problem in all universities; although almost all universities will talk about putting teaching in the first place, in the actual assessment, especially in the title assessment, it is still based on teachers' projects and papers. Therefore, it is not surprising that teachers are busy declaring projects and writing papers. “Emphasis on academics rather than teaching” is likely to lead to teachers being “perfunctory” in their teaching. Simultaneously, through supervision, it continues to deepen the reform of teaching content, methods, and means, promote teaching reform, and improve the status of the main students. Meanwhile, through field trips, student seminars, or individual interviews, it is possible to gain an in-depth understanding of whether students can receive timely and effective assistance and guidance when they encounter doubts in the learning process and to understand students' requirements and opinions on teaching materials, teaching progress, and teachers' teaching [3]. Thus, strengthening the supervision of teaching helps to detect bad teaching and learning styles among teachers and give timely correction. It creates a good campus culture [4].

### 2.4. Provide Advice and Suggestions for the Development of Teaching in the University

The teaching supervision department is an advisory body of the school, independent of the Academic Affairs Office and the teaching department. It can more objectively supervise, inspect, guide, and evaluate the whole teaching practice, give timely and objective feedback on the current teaching situation, analyze the existing problems, evaluate the quality of teaching, and put forward suggestions for improvement [5]. The teaching supervision work itself is not directly involved in management, but it can summarise the common problems in teaching through classroom listening, teaching inspection, and student seminars. The information from supervision is summarised, concluded, and analyzed in time to provide a basis for decision-making for the school's teaching department to improve teaching management and teaching staff to improve their teaching ability, such as teachers' teaching, students' learning, teaching status, teaching effect, and teaching management cooperation. It delivers timely teaching information and puts forward opinions or suggestions so that school leaders or teaching management departments can quickly grasp the teaching situation and make correct judgments and decisions. This will ensure that the teaching and learning process is standardized, orderly, and good [6].

## 3. Problems of Teaching Supervision in Applied Undergraduate Universities under the Perspective of “Internet+”

### 3.1. Emphasis on “Theory” Teaching rather than “Practice” Teaching

Whether it is the transformation of local undergraduate colleges and universities to application-oriented colleges and universities or the transformation of higher vocational high schools to application-oriented undergraduate colleges and universities, they are still in the early stage or transition stage. Applied universities cultivate application-oriented talents, which is different from academic universities and skill-oriented high vocational high schools in the past. It should be said that it cultivates both academic ideas and high-level, high-quality skill-oriented talents. Therefore, on the one hand, in the teaching supervision, we pay more attention to the teaching of theory courses than practice courses. It is a problem of the supervisors' own transformation of the idea of “application-oriented.” According to the statistics of a university's supervisors' manuals for listening and evaluating classes in the academic years of 2017-2018, 2018-2019, and 2019-2020, the proportion of listening to practical classes is 12%, 18%, and 20% respectively. On the other hand, there is a lack of perfect practical teaching evaluation standard in the teaching evaluation standard. The supervisor generally divides the practical teaching into experiment, practical training, and social practice. Therefore, the practical teaching evaluation should include these three categories. At present, the evaluation of practical teaching mostly focuses on practical operation ability, and the evaluation standard is too general to scientifically and reasonably evaluate the process and effect of practical teaching. Teaching evaluation has not yet been truly in line with the criteria for training applied talents. Therefore, using theoretical, experiment, social practice, and practical training courses targeted the form of teaching supervision [7]. In the transformation to application-oriented, how to evaluate teachers' teaching quality and strengthen the supervision of practical teaching to improve the quality of practical teaching is a topic for further research and discussion by supervisors [8]. In addition, the rapid development of “Internet+” education is bound to cause continuous reform and updating of teaching ideas, teaching modes, teaching methods, and teaching means in colleges and universities. Supervisors must adapt to the changes in educational technology and strengthen supervision of practical teaching [9]. However, at present, some universities do not pay attention to the training of teaching supervisors and do not have corresponding learning and training plans. The lack of internal and external learning and training is also an important reason why supervisors are not strong enough to supervise “practical” teaching.

### 3.2. Unstable Supervisory Team

The work of teaching supervision involves various disciplines and majors in each second-level college, and it is obviously not very realistic to have full-time supervisors corresponding to them. The small number of full-time supervisors is a common phenomenon in all universities. Especially in private universities, due to the allocation of funds, apart from a few full-time supervisors, supervisory work is mostly performed by teachers with associate or higher titles who are more senior, experienced in teaching, and responsible in the second-level colleges. Although the university also appoints secondary college supervisors for two years in general, in fact, there are cases where part-time supervisors leave their posts, and so on, to varying degrees each semester. As shown in Table 1 and Figure 1, from a review of the supervisory teams of an undergraduate university in the second semester of the 2017-2018 academic year, the 2018-2019 academic year, and the 2019-2020 academic year, the departure rate was as high as 38%. The new part-time entry was as high as 43%, with only the PE Department and the Computer Science Department having no part-time supervisory staff turnover for five consecutive semesters, with the Computer Science Department also introducing one person. Secondly, the Business Administration Department had no part-time supervisors for four semesters in two consecutive academic years, and the Logistics Department had no part-time supervisors for three consecutive semesters.

The reason for this is that, firstly, these part-time supervisors have to apply for supervisory work according to the teaching work arrangement of the second-level colleges, or they are assigned by the leaders of their departments according to their workload. Due to the high mobility of teachers in private universities, teachers' workload is not fixed every semester, sometimes more, sometimes less, and if they are responsible for part-time supervisory work when the workload is high, they will exceed the workload limit of the college. If colleges do not have additional subsidies, it will greatly reduce the motivation of part-time supervisors to participate. Secondly, part-time supervisors have to complete the teaching and research tasks of secondary colleges, then they also have to find time for supervisory management work, which is a distraction in terms of time and energy, and they are unable to cope with it, thus giving up the work of part-time supervisors. Finally, as part-time supervisors are mostly supervising and managing their own secondary colleges and monitoring their own colleagues, on the one hand, some supervisors are too harsh in their words when giving feedback afterward. On the other hand, some teachers are prejudiced against supervisors, thinking that supervision is to pick faults, so those part-time supervisors are often physically and mentally exhausted and lose their enthusiasm for supervisory work. In short, the instability of the supervisory team directly affects the consistency of the school supervisory department in listening to opinions and suggestions, the “supervision” of teachers only remains an issue, and the “guidance” becomes a mere word. This affects the continuity and effectiveness of teaching supervision.

### 3.3. Emphasis on “Supervision” rather than “Guidance”

In the work of teaching supervision, the phenomenon of emphasizing “supervision” over “guidance” is still very common, thus causing a disconnection between “supervision” and “guidance.” On the one hand, it is easier to do “supervision” than “guidance,” which is equivalent to inspection, and the results of supervision and evaluation only come from a few classroom visits [10], so it is easy to find problems, record them, and give feedback on them. However, finding out the reasons behind the problems and guiding teachers to correct them is a task that requires much effort and continuous follow-up and requires more time and energy. In reality, most supervisors prefer to give feedback in writing to the teacher's faculty leader or the teacher himself after they have found problems in the course of listening to or inspecting a class, and even if they are able to communicate face-to-face, it is only basically once, and rarely can they follow up and guide the teacher so that the teachers can move from immaturity to maturity to full maturity in the shortest possible time.

### 3.4. Single Ways and Methods of Teaching Supervision

The central part of teaching is classroom teaching activities. The level of teaching and management is reflected in classroom teaching, so the primary task of supervision is to listen to classes in-depth [11]. In terms of teaching supervision methods and approaches, at present, the traditional form of simple classroom listening and evaluation is still adopted; one or several supervisors listen to a teacher's class and then give corresponding evaluation guidance to the teacher. This is a relatively convenient way and method of supervision. However, as China's higher education progresses towards becoming an educational powerhouse and traditional undergraduate universities transform into application-oriented universities, this single way of listening to and evaluating lessons is no longer sufficient to ensure teaching quality, especially as it is difficult to conclude just one or two listening sessions. It is not always possible to conclude multiple listening sessions, and the workload of the supervisors can be very heavy, which in turn can create a very tense situation for teachers and even disrupt their teaching plans and cause resentment. In addition, in practice, some teachers do not pay attention to or rectify the feedback they receive from supervisory experts and lack motivation for teaching reform [12].

### 3.5. Lack of Integration of Teaching Evaluation Information

Although “Internet+” education has made a deep development, it does not seem to be really reflected in the field of teaching supervision work. Due to the lack of modern information technology support, the supervisors' evaluation of teachers' teaching is only retained in the paper lecture record book, and each supervisor's evaluation information is of a single-line type. If a school-level supervisor or the head of a second-level college wants to know the evaluation of a teacher by a number of supervisors for different classes, or even more so, if the teacher wants to know the information about his teaching evaluation by the supervisory institute in the past, this is undoubtedly a huge workload. At the same time, it is not easy to follow up on each teacher's evaluations as they are all messy and hidden.

## 4. Construction of Effective Teaching Supervision System of Applied Undergraduate Universities

### 4.1. Pay Attention to the Unity of Teaching Theoreticality and Practicality

In order to ensure the quality of applied talents training in private applied undergraduate colleges and universities, it is necessary to change the teaching ideas and methods that teachers used to focus only on theoretical teaching and neglect practical teaching. Thus, teaching supervision should continue to pay attention to the supervision and guidance of theoretical courses and gradually raise the requirements for practical teaching and formulate practical teaching evaluation standards. For example, whether the applicability of practical courses is reasonable, whether the hardware environment of practical teaching can serve to teach normally and effectively, and whether the teachers' attitude towards practical teaching, teaching content, and teaching effect meet the requirements of practical teaching. Quantitative and qualitative evaluation continuously improve the supervision of practical teaching and strengthen the supervision and guidance of practical teaching [13].

### 4.2. Adhere to the Part-Time Subjectivity of the Supervisory Team

Supervisors in higher education institutions are basically composed of school leaders and leaders of second-level colleges or professors. As a new private university, Guangzhou College of Technology and Business needs to build more projects and spend more money at the early stage of construction, making it difficult to set up a full-time supervisory team. In order to cut costs without affecting the smooth development of supervision work, Guangzhou College of Technology and Business has always adhered to the principle of “full-time supervision as the leader and part-time supervision as the main body” over the years. It has established a relatively stable supervision team and a relatively stable supervisory team and has shown a situation of “two high and one good.” The full-time supervisors are experts who are well versed in the laws of higher education teaching, have rich teaching experience, are impartial and healthy, and have senior associate titles or above. Part-time supervisors are professors and associate professors with rich teaching experience and profound professional foundation or lecturers with certain teaching experience and top teaching evaluation selected by each department. With the expansion of the scale of schooling, more and more professors and associate professors have been introduced to each department. At present, the number of part-time supervisors with the title of associate professor or above has reached more than 90%, which has brought the comprehensive quality of the supervisory team to a new level. Secondly, the high enthusiasm of work: most of the new private colleges and universities with the title of associate professor or above are those old teachers who have retired from public colleges and universities. The full-time and part-time supervisors are precisely the highly respected old professors selected from these people. They are often responsible, upright, and patient, and according to the arrangement of supervision work, they can all complete their tasks on time and in quality. Some even often overcomplete the task of listening to and evaluating lectures, showing high enthusiasm for their work, as shown in Table 2. Thirdly, the supervision effect is good. The biggest advantage of “part-time supervisors as the main body” is that it makes full use of teachers' resources in each department and makes up for the shortage of full-time supervisors as the focus of teaching supervision is generally on those new teachers, external teachers, or teachers with problems reflected by students. The number is often large at the beginning of the construction of private colleges and universities. The task of listening to and evaluating lessons involves various departments of the college and various specialties, which is often limited by the ability and energy of full-time supervisors alone. This allows the part-time supervisors to bring their respective professional levels into play and listen in a structured, focused, and targeted manner according to the characteristics of different disciplines and specialties in their departments, making the supervisory work more professional, distinctive, and refined. At the same time, it has also drawn the attention of each department to the teaching work and received good results. In addition, the cooperation between schools and enterprises in applied colleges and universities is getting closer and closer, and enterprises are more and more involved in the work of raising talents in colleges and universities. The enterprise element in colleges and universities is getting stronger and stronger. For this reason, introducing the evaluation standards of industrial enterprises and employing experts from industrial enterprises as teaching supervisors will evaluate teaching supervision more scientifically and reasonably [5].

### 4.3. Form a Service-Oriented Supervisory Culture Combining Supervision and Guidance

Supervision of education and teaching is a very serious task. In the past, most teachers believed that supervisors would only pick on teachers and would not praise them. Therefore, to make more teachers better accept the supervision work, the majority of supervisors must update their concepts, change the way they supervise, shift from inspection style supervision to service style supervision, and enhance their sense of service [14]. The Guangzhou College of Technology and Business Supervision Office, based on the principle of starting from the actual work of supervision, has formulated a 16-word supervision policy after careful study and discussion, namely, “summarise the experience, explore highlights, discover problems, and discuss improvement.” In the supervision, a service-oriented teaching supervision and monitoring culture with “guidance as to the main focus, supervision as the supplement, combination of supervision, and guidance to promote teaching quality through feedback” have been formed. In the practice of supervision, the 16-word policy has become the basic principle of full-time and part-time supervision. When listening to and evaluating lessons, supervisors should firstly respect teachers' supervisory philosophy of respecting the classroom and listen to and evaluate lessons from summing up experiences and digging up highlights. It is important to understand teachers through listening to lessons, summarising their teaching experience, digging out the highlights that teachers can develop sustainably, and promoting teachers' confidence in engaging in education rather than discouraging them. In educational practice, “teaching should have methods but there is no fixed method” should become the guiding ideology of supervision work to summarise the experience and explore the highlights. Secondly, the supervisory work should change its concept, insist on reform and innovation, supervise with the attitude of academic research [15], and help teachers reform their classroom teaching methods, form their own teaching style, and improve the quality of classroom teaching, based on the principle of “finding problems, discussing and improving.” When supervisors listen to classes, once they find problems, they should solve them utilizing seminars, and by discussing the problems in teaching, they should guide teachers to develop and innovate, instead of mainly criticizing to frustrate teachers' enthusiasm for teaching. In recent years, the Supervision Office has followed the 16-word supervisory principles in several types of special supervision and achieved a better supervisory effect. For example, in the supervision and evaluation of undergraduate teaching plans, we adopted the method of recommending ten teaching plans by the department, selecting the excellent teaching plans by experts, and then summarising the excellent teaching plans, in theory, to refine the core content the excellent teaching plans. Through the supervision bulletin to the whole college, thus guiding the college's educational teaching reform, especially solving the theoretical problems in lesson plan writing. Another example is that we have conducted special supervision of 30 teachers with top and bottom student evaluations in two semesters in the special evaluation of teachers' teaching. Through the supervision of the two poles of teaching evaluation, the Supervision Office formed two issues of special supervision briefs based on the experts' opinions. The first issue is a summary of the experience and supervision of outstanding teachers. It affirmed some of the teachers from the perspective of “Golden Course Teachers,” raised the teaching behaviors of outstanding teachers to a theoretical level, described the qualities of “Golden Course Teachers,” sorted out the “Golden Course Teachers” teaching behaviors, and formed an influential teaching philosophy. The newsletter is published for all young and midcareer teachers to learn from and emulate. The other issue is a supervisory briefing for teachers who have fallen behind in their evaluations. Analyzing the problems and why teachers ranked low in their evaluations helped teachers clarify their educational philosophy, establish professional ideals, enhance their professional quality, strengthen their learning from theory, and train and grow in practice. They went deep into the classroom and into practice, offering valuable solutions and suggestions on many key hot issues and weak links in teaching [16].

### 4.4. Implement a Triple Superimposed Supervision Method

Educational teaching supervision is both a policy-oriented and artistic supervision, and its supervision methods determine the quality and effect of supervision. In order to improve the coverage of supervision and create an excellent quality control culture, the Supervision Office of Guangzhou College of Technology and Business has formed a new idea in the way of supervision and innovated the way of supervision, as shown in Figure 2. It divides the traditional single supervision method into regular supervision, special supervision, and inspection supervision, realizing a triple overlay of supervision methods and receiving a good effect of comprehensive quality monitoring. Routine supervision refers to the supervision method that the Supervision Office follows up the quality of classroom teaching according to the supervision regulations of the college, and its behavior is regular, comprehensive, and universal, which is customary behavior. It mainly solves the general problems of teaching quality monitoring. The early teaching inspection focuses on the guarantee of teaching conditions, preparation for teaching, and implementation and execution of teaching tasks in each teaching unit. Midterm teaching inspection focuses on teaching and research activities, lecture listening, lesson plans, student evaluation, teaching operation, and practical teaching development in each teaching unit. The final teaching inspection focuses on teaching tasks, tutorials, Q&A, examinations, examination style, discipline, and so on. The period also includes regular and irregular inspections of classes and visits to classes by school leaders, teaching management departments, and student management departments to understand the teaching operation [17]. Special supervision refers to the special supervision carried out by the Supervision Office according to the current situation of the college's development, by understanding the problems that exist in a certain aspect of education and teaching or the experience that needs to be promoted and summarised and promoted. It conducts an in-depth and systematic understanding and deep-seated dissection of a prominent problem or highlight in teaching and learning and proposes targeted guidance through collective research and diagnosis [18]. It has the nature of timeliness, specialization, and uniqueness and is special supervision to guide the management and development of education and teaching. Inspection supervision refers to the Supervision Office, according to the work needs, under the arrangement of the board of trustees and the leadership of the college, to carry out comprehensive, partial, and special problem of education and teaching work inspection. It has the nature of supervision and guidance and is a simpler way of supervision work, such as classroom teaching order inspection and campus nurturing environment inspection. It can simply understand a certain aspect of the college and provide timely and effective supervision feedback.

### 4.5. Strengthen the Collaborative Innovation of Supervision Methods

Collaborative innovation in supervision methods is a principle that has been adhered to by the Supervision Office of Guangzhou College of Technology and Business. The innovative supervision method is proposed according to the actual construction of teachers' teams in private colleges and universities. At present, there is a common phenomenon of two more and one less in the teaching team of private colleges and universities: more retired old teachers, more new graduate students, and fewer middle-aged teachers with teaching experience; such a teacher structure poses a challenge to improve the quality of classroom teaching. In order to improve the quality of classroom teaching, let new teachers stand firmly on the podium and stand well on the podium, let veteran teachers give full play to their enthusiasm, and let young and middle-aged teachers better accumulate teaching experience; to truly play the role of classroom teaching in the education of people in the university, the College Supervision Office has changed the traditional simple mode of listening to and evaluating classes, as shown in Figure 3. It gives full play to the role of part-time supervisors and old professors to pass on, help, and lead and constantly innovates the methods of classroom teaching supervision, using “old to lead new,” “new to promote new,” “point to promote surface,” and “excellent to promote teaching,” receiving good results. In recent years, the Supervision Office has put forward three listening requirements for regular listening to lessons according to the relevance and effectiveness of part-time supervisors' listening to lessons. The first is understanding listening: listening to new teachers' lessons and external teachers' lessons to grasp the teaching dynamics of new teachers. The second is supportive listening: listening to the lessons of teachers who have been evaluated by previous students and giving precise help. The third is induction listening: listening to the lessons of new teachers so that young teachers can be competent for their posts and stand firmly on the podium. Three approaches were used in the implementation of the collaborative and innovative supervisory approach. The first is to innovate and extend the traditional form of listening and evaluating lessons by teachers on their own, in the form of a single, random lesson. For example, the PE Department has upgraded this work to include teaching and research in the same sport, with peers in the same sport communicating and evaluating the “professional competence” of their teachers in a two-way manner and judging the professional teaching ability of their peers in a realistic manner to achieve the goal of mutual learning and improvement. The second is to establish a collective work form of listening to and evaluating lessons with the teaching and research department as the main body; that is, the director of the teaching and research department takes the lead in organizing the teachers of the department to collectively listen to and evaluate the lessons of some or individual teachers with teaching characteristics. After the collective discussion and diagnosis, the teaching and research department director will designate a person to write the first draft of the collective listening report of not less than 2,000 words, which will be submitted to the part-time supervisor for review and modification. Then, the final draft will be formed after repeated modifications through collective discussion. Through this way of collective listening and evaluation activities, it can strengthen the atmosphere of scientific research and teaching and research in the teaching and research department and at the same time form a natural habit of academic thought exchange through collective discussion, which truly reflects the supervisory purpose of collaborative innovation. The third is to improve the academic analysis of young teachers, mainly in the form of listening and evaluation work, that is, the teachers who perform supervisory work from time to time to select young teachers who do not have classes, together with random listening to a teacher's classroom teaching. After listening to a class, the participating teachers discuss it with each other. Finally, the part-time supervisor or a teacher with a higher title asks questions related to the course's knowledge system and methodological system and with certain academic significance. It requires the young teachers to refine the lecturer's “shining” points according to the actual situation of the lecture they have listened to and to make constructive suggestions in a debatable tone for the shortcomings. The young teachers who have listened to the lecture will write a lecture report of at least 1500 words under the guidance of a highly qualified teacher (or supervisor). The above-mentioned innovative ways of listening to and evaluating lectures improve the teaching standard of young teachers and cultivate their academic thinking, broaden their academic vision, and enhance their academic sensitivity.

### 4.6. Establish an Information-Based Teaching Supervision and Management Platform

In order to ensure that the evaluation of teachers' teaching is scientific, objective, fair, and comprehensive, comprehensive integration of teachers' evaluation information is needed, and an evening information-based teaching supervision and management platform must be established, as shown in Figure 4. In this platform, there can be both daily and regular evaluation channels. The daily evaluation mainly includes daily evaluation of teachers by informants, daily teaching inspections, and listening to and evaluating lessons. Regular evaluation channels mainly include teaching information feedback, student evaluation symposiums, student online teaching evaluation, peer evaluation, and special teaching inspections [19]. Cloud inspection is implemented in the special supervision of special teaching materials to achieve high efficiency. All teaching materials are uploaded to the Xuexitong Cloud, and electronic versions of the materials are accessed. The preparation of teachers' teaching materials is discovered promptly through inspection, and those that are incomplete are promptly fed back into the system for rectification [20]. In this platform, the system will automatically generate a summary and aggregated evaluation of a particular teacher. Individual teachers will see all the evaluation results about themselves and will only be able to view the identity of the evaluator and not who the evaluator is. However, the results of all teachers' teaching evaluations are only available to individuals; for example, general supervisors can only see the evaluations of their peer supervisors, and school-level supervisors can see everyone's evaluations. Here, teachers' privacy can be ensured, while the information of teachers' teaching evaluation can be integrated and summarised, effectively ensuring the scientific, fair, and authoritative teaching supervision and evaluation results. At the same time, within the information management platform, there will also be a record of the supervisor's follow-up guidance to teachers so that the “guidance” to teachers can be traced and documented, thus ensuring the effectiveness of supervision. Therefore, teaching supervision departments should speed up the construction of information technology and develop an information-based teaching supervision management platform suitable for their own schools to escort the creation of a high-level applied university.

## 5. Conclusion

This paper expounds the significance of teaching supervision and describes the problems in the teaching of “Internet plus” supervision, as shown in Table 1. From 2017 to 2020, the number of types of resignation supervision has reached more than 30%. As shown in Table 2, in the 2019-2020 academic year, 25 part-time supervisors attend 2856 classes a year, with 32 teaching weeks a year, with an average of 114.24 class hours per supervisor per year. Therefore, it constructs the teaching supervision system of application-oriented undergraduate colleges and universities.

With the rapid development of “Internet +” and the application-oriented and efficient transformation, it is very necessary to build an effective teaching supervision system. The follow-up research will focus on the following aspects:

1. Establish an information-based teaching supervision and management platform to facilitate the development of supervision work.
2. The supervision mode of triple superposition is implemented in practice, and the work is clear.
3. Strengthen the subjective role of part-time supervision and coordinate the synchronization of part-time supervision in supervision and teaching.

In the future, the rapid development of informatization will further promote the development of teaching supervision towards more scientific, standardized, and convenient. As a supervision department, especially the managers and supervisors of the supervision department, they should also constantly update their supervision concept, strengthen their service awareness, establish a model, give full play to their supervision and guidance role, become a bridge between the school management organization and teachers and students, so that the supervision work can better serve the school and teachers and students, benefit from the school, and finally improve the education and teaching quality of the school.

## Figures and Tables

**Figure 1:** Proportion of part-time supervisors leaving/recruiting.

**Figure 2:** The triple stacked supervision approach.

**Figure 3:** Collaborative and innovative approach to supervision.

**Figure 4:** Functions of the information-based teaching supervision management platform.

**Table 1:** Turnover of part-time supervisors.

Department	Academic year														
	2017-2018-2			2018-2019-1			2018-2019-2			2019-2020-1			2019-2020-2		
	Situation														
	On duty	Leaving post	Recruitment	On duty	Leaving post	Recruitment	On duty	Leaving post	Recruitment	On duty	Leaving post	Recruitment	On duty	Leaving post	Recruitment
Department of Economy	2	0	0	4	1	3	4	0	0	3	1	0	3	0	0
Department of Electronic Studies	2	2	2	2	2	2	2	1	1	2	0	0	2	1	1
Department of Music	1	0	0	1	1	1	1	1	1	1	0	0	1	1	1
Department of Foreign Languages	2	1	1	0	2	0	0	0	0	2	0	2	2	0	0
Accounting Department	2	1	1	2	0	0	4	0	2	4	1	1	3	1	0
Department of Business and Administration	2	0	0	2	0	0	2	0	0	3	1	2	2	1	1
Department of Fine Arts	1	1	1	1	0	0	1	0	0	2	1	2	1	1	0
Logistics Department	3	0	0	3	0	0	3	2	2	2	1	0	2	0	0
Computer Department	2	0	0	3	0	1	3	0	0	3	0	0	3	0	0
Department of Physical Education	1	0	0	1	0	0	1	0	0	1	0	0	1	0	0
Department of Basic Courses	1	1	1	1	1	1	1	0	0	1	1	1	2	1	2
Ideological and Political Department	1	1	1	1	1	1	1	0	0	0	1	0	0	0	0
Total	20	7	7	21	8	9	23	4	6	24	7	8	22	6	5

**Table 2:** Attendance statistics for full-time and part-time supervisors, 2018–2020.

Academic year	Number of lectures	Semester 1	Semester 2	Total lectures (section)
2018-2019	27	1089	1269	2358
2019-2020	25	1470	1386	2856

## Data Availability

The experimental data used to support the findings of this study are available from the corresponding author upon request.
